# A GRU-Based Method for Predicting Intention of Aerial Targets

**DOI:** 10.1155/2021/6082242

**Published:** 2021-11-02

**Authors:** Fei Teng, Yafei Song, Gang Wang, Peng Zhang, Liuxing Wang, Zongteng Zhang

**Affiliations:** ^1^Air and Missile Defense College, Air Force Engineering University, Xi'an 710051, China; ^2^AVIC Jiangxi Hongdu Aviation Industry Group Company Ltd., Nanchang 330024, China

## Abstract

Since a target's operational intention in air combat is realized by a series of tactical maneuvers, its state presents the characteristics of temporal and dynamic changes. Depending only on a single moment to take inference, the traditional combat intention recognition method is neither scientific nor effective enough. Based on a gated recurrent unit (GRU), a bidirectional propagation mechanism and attention mechanism are introduced in a proposed aerial target combat intention recognition method. The proposed method constructs an air combat intention characteristic set through a hierarchical approach, encodes into numeric time-series characteristics, and encapsulates domain expert knowledge and experience in labels. It uses a bidirectional gated recurrent units (BiGRU) network for deep learning of air combat characteristics and adaptively assigns characteristic weights using an attention mechanism to improve the accuracy of aerial target combat intention recognition. In order to further shorten the time for intention recognition and with a certain predictive effect, an air combat characteristic prediction module is introduced before intention recognition to establish the mapping relationship between predicted characteristics and combat intention types. Simulation experiments show that the proposed model can predict enemy aerial target combat intention one sampling point ahead of time based on 89.7% intent recognition accuracy, which has reference value and theoretical significance for assisting decision-making in real-time intention recognition.

## 1. Introduction

With the development of military and aviation technology, informationization has gradually become the focus of the modern battlefield. Information-driven has become the main direction of modern war. As technological development and application have led to a dramatic increase in the amount of battlefield information, it has become difficult to recognize the enemy's intention from multiple sources of battlefield data in a timely and effective manner by relying solely on the experience of domain experts. There is a need for intelligent methods to eliminate the drawbacks of manual methods [1, 2].

To meet the needs of operational decision systems, many intention recognition studies have been conducted. Research on enemy target operational intent recognition mainly includes methods such as evidence theory [3, 4], template matching [5, 6], expert systems [7], Bayesian networks [8, 9], and neural networks [2, 10–12]. Past research [2–12] has achieved enemy target operational intention recognition according to different operational contexts, but there are shortcomings in temporal characteristic learning and knowledge representation. On the one hand, the target operational intention is realized through a series of tactical maneuvers, so the dynamic attributes of the target and the battlefield environment will change over time. In addition, the enemy target has a certain degree of concealment and deception when performing combat operations. Thus, the above methods are not scientific enough as they determine the enemy target operational intention using characteristic information at a single moment. On the other hand, the above methods require explicit organization, abstraction, and description of military experts' empirical knowledge, so the knowledge representation and engineering implementation are difficult. Aiming at the drawbacks of the above methods, Ou et al. [13] proposed an intelligent recognition model of tactical intention based on a long short-term memory (LSTM) network. The input characteristic of the model is 12 consecutive frames of time sequence characteristics, which can effectively overcome the judgment by a single moment. Moreover, the model implicitly organizes, abstracts, and describes the empirical knowledge of military experts, making its knowledge representation and engineering implementation less difficult. However, it only uses historical moment information to make inferences about current information and cannot effectively use future moment information. Since there are many characteristics related to the intention of air targets, it is necessary to highlight the influence of key characteristics and reduce the contribution of redundant characteristics. In addition, we want to further improve the real-time performance of aerial target intent recognition in some way.

Based on the above analysis, we propose a gated recurrent unit (GRU) based intelligent prediction model for aerial target combat intention. The model has characteristic prediction and intention recognition modules. The intention recognition module introduces a bidirectional propagation mechanism, attention mechanism, and particle swarm optimization (PSO) algorithm based on a GRU to build an intelligent intention recognition model. With similar performance to that of LSTM, a GRU has less structural complexity and requires less time for recognition. Compared with a GRU, a bidirectional gated recurrent unit (BiGRU) can use not only the information of historical moments but also that of future moments to make comprehensive judgments. PSO can find the optimal parameters of a BiGRU network [14], and the attention mechanism layer can further highlight the key information affecting the intention and improve the accuracy of intention recognition. In order to realize our idea of further shortening the time used for intention recognition, we build a characteristic prediction module that uses the BiGRU network to analyze the collective characteristics and predicts future aerial target characteristics, which are input to the intention recognition module to establish the mapping relationship between future aerial target characteristics and the target's operational intention types. Experiments show that the proposed model can predict the enemy aerial target operational intention one sampling point in advance, and the accuracy rate is increased by 2.9% compared with LSTM.

The remaining sections of this paper are arranged as follows.  Section 2 introduces the definition of intent recognition of aerial targets and how to select intention categories and characteristic types. In Section 3, the framework of the proposed model is described in detail, including the intention recognition module and the characteristic prediction module. Experimental results are analyzed in Section 4 to show the performance of the new method. This paper is concluded in the last section.

## 2. Description of Aerial Target Operational Intention Recognition Problem

Intention recognition is important for command and control in modern war. The operational intention of aerial target can be inferred based on real-time data from multiple sensors in a dynamic and complex battlefield environment. To enhance the reliability of intention recognition, a priori knowledge and the experience of experts in the relevant operational field [12] should also be taken into consideration. The process of intention recognition is shown in Figure 1.

Aerial target intention recognition is a pattern recognition problem that can be described as a mapping of intention recognition characteristics to aerial target combat intention types. Define the vector **V**^(*t*)^ as the real-time air combat characteristic information at time *t* and **P**=(*p*_1_, *p*_2_,…, *p*_*n*_) as the aerial target combat intention space set. Due to the complexity, high confrontation, and deceptive nature of actual air combat environment conditions, relying on the real-time air combat characteristic information detected at a single time can be somewhat deceptive and one-sided. To infer the combat intention of an enemy aircraft from air combat characteristic information at successive times is far more accurate and scientific than to rely on information at a single time [1]. The mapping function from the space set **P** of operational intention to the temporal characteristic set **V**_*m*_ is determined by defining **V**_*m*_ as the temporal characteristic set for *m* consecutive moments from *t*_1_ to *t*_*m*_:

(1) $$\begin{array}{c} P=f\left(V_{m}\right)=f\left(V^{\left(t_{1}\right)},V^{\left(t_{2}\right)},\ldots ,V^{\left(t_{m}\right)}\right). \end{array}$$

It can be seen that to achieve accurate recognition of the operational intention of aerial targets requires a combination of professional military knowledge and operational experience and complex thinking activities such as extraction, comparison, analysis, association, and inference of key information of air warfare. It is difficult to establish the mapping relationship between **V**_*m*_ and **P** by a single formula [13]. We implicitly establish the mapping relationship between the characteristic set and operational intention by training bidirectional gated recurrent units with attention mechanism (BiGRU-Attention) network structure using an aerial target operational intention recognition characteristic set.

### 2.1. Description of Space Set of Aerial Target Operational Intention

The target operational intention space set varies for different operational forms, enemy entities, and desired contexts. Therefore, the operational intention space set of enemy targets must be defined based on the corresponding operational context, attributes of the enemy targets, and possible operational tasks. For example, a target intention space set was established as {avoidance, patrol, attack} based on the potential threat of underwater targets [15]; an operational intention space set was established as {retreat, cover, attack, reconnaissance} for a single group of enemy maritime ship formations [16]; and an operational intention space set of aerial targets was defined as {reconnaissance, surveillance, attack, penetration} [17]. By taking UAV close-range engagement as the research object, we establish the combat intention space set of enemy targets as seven types of intention, {feint, surveillance, electronic interference, penetration, attack, retreat, reconnaissance}.

After determining the space set of enemy operational intention, the key to applying the proposed intelligent recognition model is to convert human cognitive models to labels that can be trained by intelligent models and which correspond to the types of intention in the operational intention space set [18]. The cognitive experience of experts at air warfare can be encapsulated in labels to train the model. A set of label values {0, 1, 2, 3, 4, 5, 6} is set for the intention types in the established combat intention space set.  Figure 2 shows the corresponding combat intention type coding and model resolution mechanisms. For example, if the intention prediction result is 5, then the combat intention of the enemy target against our target is retreat. Therefore, this knowledge encapsulation and model parsing can clearly and easily describe human empirical knowledge and facilitate model training.

### 2.2. Selection of Aerial Target Combat Intention Characteristic

The enemy aerial target's operational intention is highly correlated with its operational mission, the mutual threat level between the two sides, and the tactical maneuvers. According to the abovementioned three aspects and the requirement of easy acquisition by radar, the characteristics that are closely related to the combat intention of the air target are selected.

Analyzed from the perspective of operational tasks, when an enemy UAV performs a certain task, enemy aircraft characteristics must meet certain conditions. For example, when performing defense penetration tasks, it is divided into high-altitude penetration and low-altitude penetration, and the corresponding heights are 10 ~ 11 km and 100 m ~ 1000 m; a high flight speed of fighter aircraft when receiving attacks is generally 735 ~ 1470 km/h [12]. There is also a connection between the aerial target radar signal status and the combat mission. A fighter usually turns on air-to-air radar and electronic jamming in air combat, and marine radar and air-to-air radar on a reconnaissance mission [19].

Many factors affect the threat level between the two targets. For convenient experimental data collection, we consider the speed, flight acceleration, distance, flight altitude, heading angle, and azimuth angle of both the enemy's and our warplanes [20], as shown in Figure 3.

The air combat capability factor [21] affects the target threat level. For fighter aircraft, a single aircraft air combat capability threat function is constructed as

(2) $$\begin{array}{c} C=\left[\ln\;\varepsilon_{1}+\ln\left(\varepsilon_{2}+1\right)+\ln\left(\sum \varepsilon_{3}+1\right)\right]\varepsilon_{4}\varepsilon_{5}\varepsilon_{6}\varepsilon_{7}, \end{array}$$

where *ε*_1_ ~ *ε*_7_ are parameters of warplane maneuverability, airborne weapon performance, airborne detection capability, warplane operational performance, warplane survivability, warplane operational range, and electronic information countermeasure capability, respectively. The air combat capability factors of various warplanes of both sides can be calculated through this formula for a certain period of time and are saved in the database and updated at any time according to current information [22].

The realization of the operational intention of the aerial target is closely related to the maneuvers of the aircraft. There are two kinds of maneuver libraries in common use: the typical tactical maneuver library and the basic maneuver library. Since this paper studies intention recognition based on temporal characteristics, target combat intention recognition is carried out using 12 consecutive momentary characteristics as a sample. However, the control algorithm of a typical tactical action library is complicated to solve, and the exit and conversion time nodes of a maneuver are difficult to determine. The traditional basic maneuver library [23] includes only seven maneuvers, and the combined maneuvers are not rich enough. They all adopt the limit maneuver, which is inconsistent with the actual air combat situation. We adopt an improved basic maneuver library [24] that includes 11 maneuvers {left turn, right turn, accelerated forward flight, even-speed forward flight, decelerated forward flight, climb, left climb, right climb, dive, left dive, right dive}.

In summary, we use an aerial target combat intention characteristic consisting of a 16-dimensional characteristic vector of {enemy aircraft flight altitude, our aircraft altitude, enemy aircraft flight speed, our aircraft flight speed, enemy aircraft acceleration, our aircraft acceleration, enemy aircraft air combat capability factor, our aircraft air combat capability factor, heading angle, the distance between the two sides, azimuth angle, air-to-air radar status, marine radar status, maneuver type, jamming status, jammed status}, which can be divided into numeric and nonnumeric characteristics, as shown in Figure 4.

## 3. Model Framework

The proposed aerial target operational intention prediction model consists of a characteristic prediction module and an intention recognition module, as shown in Figure 5. The characteristic prediction module is based on the BiGRU network. The historical aerial target operational intention recognition characteristic set **V**_*m*_ is used as input, a linear default activation function of the fully connected layer is used to obtain the prediction characteristic set **W**_*m*_, and these two sets are formed into the temporal characteristic data and input to the intention recognition module constructed by the BiGRU-Attention [25] network. The probability of each intention type is calculated using the softmax function, and the maximum probability intention type label is output as the aerial target combat intention recognition result. The characteristic prediction module and intention recognition module are described below.

### 3.1. Characteristic Prediction Module

The BiGRU characteristic prediction module has three parts: the aerial target combat intention characteristic set input layer, hidden layer, and output layer. Reference [26] has confirmed that the prediction accuracy of each feature independently is higher than the overall prediction accuracy. Thus, Input = (Number of samples,8,1), where 8 is the time step and 1 is the characteristic dimension; and Output = 1; that is, the output characteristic dimension is 1. The detailed description will be given below.

#### 3.1.1. Input Layer

The input layer preprocesses the collected aerial target characteristic dataset into a vector form that can be accepted and processed by the BiGRU layer, as follows:

(1) Read the dataset and clean the data.
(2) Code nonnumeric data of jamming state, jammed state, air-to-air radar state, and marine radar state as 0 (off) or 1 (on). Millier's nine-level quantization theory [27] is used to quantize numeric data of maneuver types.
(3) Normalize encoded nonnumeric data with numeric data, so as to improve network convergence speed and accuracy and prevent model gradient explosion. We normalize 11 types of numeric data and five types of encoded nonnumeric data. For the *i*th dimensional characteristic data, **G**_*i*_=[*g*_*i*1_, *g*_*i*2_,…, *g*_*ix*_,…, *g*_*in*_],  *i*=1,2, ⋯，16, where *n* is the total number of data points. *g*_*ix*_′ is the result of normalizing the *x*th original data of the *i*th dimensional characteristic to [0, 1]; that is,
  (3) $$\begin{array}{c} g_{ix}^{\prime }=\frac{g_{ix}-\min G_{i}}{\max G_{i}-\min G_{i}}, \end{array}$$
where max**G**_*i*_ and min**G**_*i*_ are the maximum and minimum values, respectively, of **G**_*i*_.
(4) Divide the data into training and test sets at an 8 : 2 ratio
(5) Construct training and test samples as follows. Using the method of predicting a single characteristic in turn, take the distance characteristic prediction of the enemy and ourselves as an example. If the distance data of the 1∼8 moments are used to predict the distance *D*_9_ at moment ninth, the function mapping relationship is
  (4) $$\begin{array}{c} D_{9}=f\left(d_{1},d_{2},\ldots ,d_{8}\right),\; \end{array}$$
where *d*_*i*_, *i* ∈ (1,2 ⋯ , 8) is the distance at the *i*th moment. *d*_1_ ~ *d*_8_ are selected as the first set of input data, labeled as *d*_9_; *d*_2_ ~ *d*_9_ are selected as the input data, labeled as *d*_10_, and so on. The training sample input data and training sample labels are generated this way and shown below. The test data are constructed in the same way as the training sample data [28].

(5) $$\begin{array}{c} \left[\begin{array}{cccc} d_{1} & d_{2} & \cdots & d_{m}\\ d_{2} & d_{3} & \cdots & d_{m+1}\\ \vdots & \vdots & \ddots & \vdots \\ d_{8} & d_{9} & \cdots & d_{m+7} \end{array}\right],\\ \left[\begin{array}{cccc} d_{9} & d_{10} & \cdots & d_{m+8} \end{array}\right]. \end{array}$$

The collected aerial target combat intention characteristic set **V**_*m*_ is now in a characteristic vector form that can be directly accepted and processed by the hidden layer.

#### 3.1.2. Hidden Layer

As a variant of the recurrent neural network (RNN), a gated recurrent unit (GRU) [29] has a similar recursive structure and a memory function to process time-series data. A GRU can alleviate the problems of gradient disappearance and explosion that may occur during RNN training, thus solving the long-term memory problem. Another RNN variant, the long short-term memory (LSTM) network [30], performs similarly, but a GRU has a simpler structure and can reduce computation and improve training efficiency.

Figure 6 shows the internal structure of the GRU. Its two inputs are the output state **h**_*t*−1_ at the previous moment and the input sequence value **x**_*t*_ at the current moment, and the output is the state **h**_*t*_ at the current moment. It updates the model state through two gates. The reset gate **r**_*t*_ controls the degree of forgetting the historical state information so that the network can discard unimportant information, and the update gate **z**_*t*_ controls the weight of the previous moment's state information being brought into the current state, helping the network to remember long-time information [31]. These variables are related as follows:

(6) $$\begin{array}{c} \left\{\begin{array}{c} r_{t}=\sigma \left(W_{r}x_{t}+U_{r}h_{t-1}\right),\\ z_{t}=\sigma \left(W_{z}x_{t}+U_{z}h_{t-1}\right),\\ {\tilde{h}}_{t}=\tan\text{h}\left(W_{\tilde{h}}x_{t}+U_{\tilde{h}}\left(r_{t}⊙h_{t-1}\right)\right),\\ h_{t}=\left(1-z_{t}\right)⊙h_{t-1}+z_{t}⊙{\tilde{h}}_{t}, \end{array}\right) \end{array}$$

where *σ* is the sigmoid activation function, which transforms the intermediate states into the range [0,1]; **h**_*t*−1_ and **h**_*t*_ are output states at time *t* − 1 and *t*, respectively; **x**_*t*_ is the input sequence value at time *t*; ${\tilde{h}}_{t}$ is the candidate output state; **W**_*r*_, **W**_*z*_, $W_{\tilde{h}}$, **U**_*r*_, **U**_*z*_, and $U_{\tilde{h}}$ are weight coefficients corresponding to each component; tanh is the hyperbolic tangent function; and ⊙  is the Hadamard product.

The traditional GRU structure propagates unidirectionally along the sequence transmission direction, and it acquires historical information before the current moment, ignoring future information. BiGRU, as shown in Figure 7, includes a forward and backward GRU, which can capture the characteristics of the information before and after the current moment [32]. In Figure 7, GRU^1^ is a forward GRU and GRU^2^ is a backward GRU. The output state **h**_*t*_ of BiGRU at moment *t* can be obtained from the forward output state ${\overset{⟶}{h}}_{t}$, determined by the input **x**_*t*_ at moment *t* and output state ${\overset{⟶}{h}}_{t-1}$ of the forward GRU at moment *t*−1, and the backward output state ${\overset{\leftarrow }{h}}_{t}$, determined by the input **x**_*t*_ at moment *t* and output state ${\overset{⟶}{h}}_{t+1}$ of the backward GRU at moment *t* + 1.

#### 3.1.3. Output Layer

The output **h**_*t*_ of the BiGRU network in the hidden layer is fed to the fully connected layer in the output layer, and the final prediction characteristic values are output using a linear activation function.

### 3.2. Intention Recognition Module

The BiGRU-Attention intention recognition module has input, hidden, and output layers. The hidden layer has BiGRU and Attention mechanism layers. In the network, the Input = (Number of samples,12,16), and the Output = 7, where 12 denotes the time step, 16 denotes the number of characteristic dimensions, and 7 denotes the total number of intention types. The detailed description will be given below.

#### 3.2.1. Input Layer

The input layer of the characteristic prediction module has cleaned and normalized the collected aerial target operational intention characteristics, so the intention recognize module input layer is mainly for the construction of the sample data of the intention recognition module. If the characteristic data of the 1∼12 moments are used to predict the intention during that time, the function mapping relationship is

(7) $$\begin{array}{c} Q_{1}=f\left(v_{1},v_{2},\ldots ,v_{11},w_{12}\right),\; \end{array}$$

where *Q*_1_ denotes the prediction intention types in time periods 1∼12; **v**_*i*_, *i* ∈ (1,2,…, 11) denotes the historical characteristic data at moment *i*, and **w**_12_ denotes the characteristic data predicted by the characteristic prediction module at moment 12.  (**v**_1_, **v**_2_,…, **v**_11_, **v**_12_) is the first set of input data, labeled as intention type *q*_1_ corresponding to time periods 1∼12; (**v**_2_, **v**_3_,…, **v**_12_, **v**_13_) is the second set of input data, labeled as the intention type *q*_2_ corresponding to time periods 2∼13, and so on. The training sample input data and labels are composed as shown below. The test and training sample data are constructed similarly, except the former replaces the characteristic **v**_*t*_ at the last moment of each sample with the characteristic **w**_*t*_ predicted by the characteristic prediction module; that is, the input data are (**v**_*i*_, **v**_*i*+1_,…, **v**_*i*+10_, **w**_*i*+11_), and the label is the intention type *q*_*i*_ corresponding to the time period *i* ∼ *i* + 11.

(8) $$\begin{array}{c} \left[\begin{array}{cccc} v_{1} & v_{2} & \cdots & v_{m}\\ v_{2} & v_{3} & \cdots & v_{m+1}\\ \vdots & \vdots & \ddots & \vdots \\ v_{11} & v_{12} & \cdots & v_{m+10}\\ v_{12} & v_{13} & \cdots & v_{m+11} \end{array}\right],\\ \left[\begin{array}{cccc} \;q_{1}\; & q_{2} & \;\cdots \; & q_{m} \end{array}\right]. \end{array}$$

After one-hot encoding of the intention labels, it is sent to the hidden layer together with the constructed sample data.

#### 3.2.2. Hidden Layer

The hidden layer contains the BiGRU network layer and attention mechanism layer. The BiGRU layer has been described. The attention mechanism layer is described below. The attention mechanism [33–35] operates similarly to the human brain by focusing on the local content of an object according to its purpose. The attention mechanism highlights characteristics that account for a greater proportion of prediction results by calculating the weights of characteristic vectors output from the BiGRU network at different moments. In aerial target combat intention recognition, the neural network assigns weight coefficients so as to focus on some key characteristics during the training process through the attention mechanism. Its implementation is to learn the importance of each characteristic and then assign the corresponding weight coefficient according to its importance. For example, if an enemy aircraft executes a penetration, its flight altitude and heading angle will be assigned higher weights. The structure of the attention mechanism model is shown in Figure 8.

The characteristic vector **h**_*t*_ output by the BiGRU network at moment *t* is input to the attention mechanism layer to obtain the initial state vector **S**_*t*_. Learn the initialization vector **e**_*t*_ of the attention mechanism by equation (9), and the attention weights are probability by equation (10), i.e., the softmax function, to obtain the weight probability vector *α*_*t*_. The final state vector **Y** is obtained by equation (11) [36]. The formula is as follows:

(9) $$\begin{array}{c} e_{t}=\tan\;h\left(W_{w}S_{t}+b_{w}\right), \end{array}$$

(10) $$\begin{array}{c} \alpha_{t}=\frac{\exp\left(e_{t}u_{w}\right)}{\sum_{i=1}^{t}\left(e_{t}u_{w}\right)}, \end{array}$$

(11) $$\begin{array}{c} Y=\sum_{t=1}^{n}\alpha_{t}S_{t}, \end{array}$$

where **W**_*w*_ is the weight coefficient matrix, **b**_*w*_ is the bias coefficient matrix, and **u**_*w*_ is a matrix vector initialized randomly and continuously learning with training.

#### 3.2.3. Output Layer

The output of the attention mechanism layer is fed into the multiclassification activation softmax function, which outputs the label with the highest probability of aerial target combat intention. The enemy aerial target combat intention can be recognized by parsing the label, as in Figure 2. The output prediction label is

(12) $$\begin{array}{c} y_{k}=\text{softmax}\left(WY+b\right), \end{array}$$

where **W** is the weight coefficient matrix with training, **b** is the corresponding bias matrix, and  *y*_*k*_ is the predicted label of the output.

## 4. Experimental Analysis

### 4.1. Experimental Dataset and Environment

This experiment took an airspace UAV close-range engagement as the research background, and the experimental data were extracted from a combat simulation system. Using the characteristic processing and coding described in this paper, the state characteristics of 12 consecutive frames of the enemy aerial target were collected for each sample [13], where 10,000 samples (8,000 training and 2,000 testing) were constructed, including 16 pieces of information, such as flight speed, flight altitude, azimuth, and jamming status, as characteristics. Due to a large amount of data in the sample set, intention-type labels were generated by computer according to the rules, and experts corrected data with intention classification ambiguity. Dataset labels included seven intention types, and the combat intention data consisted of 11.8% surveillance, 14.65% reconnaissance, 18.15% feint, 18% attack, 13.9% surprise, 12.3% retreat, and 11.2% electronic jamming.

We used Python 3.8 on a Quadro RTX 5000/PCle/SSE2 GPU with CUDA 11.0 acceleration environment, with a Keras 2.4.3 deep learning framework and an x86-64 CentOS7 PC system, Intel® Xeon® Sliver 4110 CPU @2.10 GHz, and 64 GB RAM.

### 4.2. Experimental Analysis of Characteristic Prediction Module

The task of the characteristic prediction module is to predict the future characteristics of enemy aerial targets, which are later input to the intent recognition module to predict enemy aerial target intent. The average of the mean square error (which we will refer to as “error”) of 16-dimensional features was used as the evaluation index.

#### 4.2.1. Network Structure Selection

The network structure mainly sets the time step, number of hidden layers, and number of hidden layer nodes. Since an increased number of hidden layers will rapidly increase the time cost, considering the high requirement of air warfare on timeliness, it was set to a single or double hidden layer structure without considering more hidden layers. The results of the time step selection and hidden layer node number selection experiments are shown in Figure 9.

From Figure 9, it can be seen that the mean value of the prediction mean square error was smallest when the time step was 8, and the mean value of the prediction mean square error was smallest when the number of nodes in the single hidden layer was 18. Therefore, a network structure with a time step of 8, a single hidden layer, and 18 network nodes was chosen. The optimizer was Adam [37], the initial learning rate was 0.001; the decay rate was 0.9, the training epochs were 100, and the batch size was 512.

#### 4.2.2. Comparison Experiment

To verify that the proposed characteristic prediction module was effective and efficient, it was compared with the RNN [38], LSTM [39], GRU [40], and BiLSTM networks in terms of both real time and mean square error, and a segment of the predicted trajectory with the characteristic of the distance between the two enemy sides was selected for comparison with the actual trajectory. The results are shown in Table 1 and Figure 10.

From Table 1, we can see that BiLSTM had the longest single-step prediction time, 0.311 ms, and RNN had the shortest single-step prediction time, but its prediction error was larger, reaching 8.14 × 10^−5^. BiGRU had the smallest prediction error, and its single-step prediction time decreased by about one-third compared with BiLSTM, so it can be concluded that BiGRU had less internal structure complexity [41], with similar or even better performance than BiLSTM. The prediction error of BiGRU was half that of GRU, and it can be concluded that the bidirectional propagation mechanism could more effectively utilize the information of future moments than the one-way propagation. Although BiGRU had a longer single-step prediction time than GRU, the single-step prediction time of 0.202 ms is sufficient to provide timely prediction information when the sampling interval is 0.5s. It can be seen from Figure 10 that the characteristic trajectories predicted by RNN had a low fit to the actual characteristic trajectories, and those predicted by the other four methods had a high fit, which is consistent with the error results in Table 1.

### 4.3. Experimental Analysis of Intention Recognition Module

The data used in this experiment did not contain future characteristics predicted by the characteristic prediction module; that is, the 12 frames of temporal characteristics in each sample were all historical, with no added prediction characteristics. The purpose of the experiment was to compare our methods with those proposed in other literatures. The intention prediction experiment is described in Section 4.4.

#### 4.3.1. Network Structure Selection

The optimal network structure of BiGRU was selected using PSO [42] with four parameters: number of hidden layers, number of hidden layer nodes, batch size, and learning rate. The upper and lower limits were set as [4,500,1000,0.005] and [1,10,100,0.0001]. The intention recognition error rate was set as the fitness function, the maximum number of iterations was 20, and the population size was 30. The experimental results and settings of other key hyperparameters are shown in Table 2.

#### 4.3.2. Analysis of Intention Recognition Results

The BiGRU-Attention intention recognition module was trained and then the test samples were input into the module. The experiment showed that the accuracy of the proposed intention recognition network model proposed was achieved. To further observe the relationship between the recognition intentions, a confusion matrix of the intention recognition results of the test samples was produced. The diagonal line indicates the number of correctly recognized samples, and the results are shown in Figure 11.

It can be seen from Figure 11 that the BiGRU-Attention intention recognition model had a high recognition accuracy and recall rate for all seven intentions. In particular, the electronic interference intention recognition precision and recall rate could reach 100% and 96%, respectively. A few cases of mutual recognition errors occurred between surveillance and reconnaissance intentions and between feint and attack intentions, which should be attributed to the high characteristic similarity and deception between the intention pairs, causing the model trained by BiGRU-Attention model to have similar weights for the two intentions in each pair. As a result, the attention layer failed to accurately sense the weight difference between the two intentions, leading to a small number of incorrectly recognized intentions, which accords with the actual situation.

#### 4.3.3. Comparison Experiments

In the experiment, the highest accuracy of the test set during 200 iterations was selected as the accuracy of the intention recognition model, and the corresponding loss value was the loss value. The BiGRU-Attention intention recognition model was compared with the LSTM-based tactical intention recognition model for the battlefield against enemy targets [13], the aerial target combat intention recognition model using the Adam algorithm and ReLU function optimized DBP neural network [12], and the stacked self-encoder tactical intention intelligent recognition model [15]. The parameters of the comparison experiments were set as shown in Table 3, and the experimental results are shown in Table 4.

As can be seen from Table 4, the BiGRU-Attention intention recognition model was superior to the other three models in terms of both accuracy and loss value, with 2.5% improvement in accuracy over LSTM, and nearly 10% over SAE and DBP, thus verifying its effectiveness for aerial target combat intention recognition. Further analysis shows that BiGRU-Attention and LSTM, as temporal characteristic networks based on recurrent neural networks, were more applicable to aerial target combat intention recognition than the other two models, further indicating that it is more scientific to make inferences about aerial target combat intention based on temporal characteristic changes.

#### 4.3.4. Ablation Experiments

Although the BiGRU-Attention intention recognition model has been validated in comparison experiments for its effectiveness in operational intention recognition of aerial targets, the comparison method is not a comparison of hybrid experimental models of the same type. Results of ablation experiments on the same dataset are shown in Table 5 and Figure 12.

From Table 5, the BiGRU-Attention intention recognition model had an accuracy 2.7%, 1.9%, and 1.6% percentages higher than the accuracy of the GRU, BiGRU, and GRU-attention intention recognition models, respectively. The BiGRU-Attention model also had lower loss values than the other models. BiGRU and GRU-Attention models have similar accuracy and loss values and are better than GRU models. From Figure 12, we can see that the accuracy of the four models increased and the loss value decreased with the number of training epochs; the accuracy and loss value of the BiGRU-Attention and BiGRU models converged at around 50 rounds, and the other two models at about 70 rounds, so the introduction of bidirectional propagation seems to have effectively improved model convergence and accelerated learning. The curves of the BiGRU-Attention model were significantly better than those of the other three. The accuracy and loss curve of the BiGRU and GRU-Attention models after convergence are similar, and they are better than the GRU model, which shows that the basic GRU model was significantly improved by introducing the attention mechanism and bidirectional propagation mechanism.

### 4.4. Experimental Analysis of Intention Prediction

This experiment combined future characteristic states predicted by the characteristic prediction module and historical characteristic states into 12 frames of temporal characteristics; that is, the first 11 frames were historical characteristics, the 12th was predicted future characteristics, and sample data were constructed as described in Section 3.1.

To verify that the proposed intention prediction method can effectively recognize the enemy's intention in advance, it was compared with the intention recognition method in Section 5, which has no prediction effect, and the model evaluation indicators of precision rate, recall rate, and F1-score were used to verify the model, with results as shown in Table 6 and Figure 13.

From Table 6 and Figure 13, the proposed intention prediction method had high prediction accuracy for retreat and electronic jamming intentions, but relatively low accuracy for surveillance and attack intention recognition. After analysis, the air combat characteristics of the first two intentions were more obvious, and the air combat characteristics of the latter two intentions were more similar to those of the reconnaissance and feint intentions, which causes mutual prediction error that results in relatively low accuracy of intention prediction. Overall, the accuracy of the proposed intention prediction method could reach 89.7%, which is a significant improvement in accuracy compared with LSTM, DBP, and SAE, and could produce the prediction one sampling interval (0.5 s) earlier.

In addition, the attempt to predict the enemy's intention in advance of two sampling points did not yield satisfactory results, and the accuracy could only reach 70%. Compared with single-step prediction, the two-step prediction of the characteristic prediction module has too much error accumulation, and the goodness of fit is low, which leads to the low accuracy of intention prediction. However, with the continued development and improvement of multistep prediction methods, it is believed that the proposed aerial target combat intention prediction method can have better application prospects.

## 5. Conclusions

For the problem of aerial target combat intention recognition, we adopted a hierarchical strategy to select 16-dimensional air combat characteristics from three perspectives: enemy combat mission, threat level between two sides, and tactical maneuvers. The sample vector is constructed by preprocessing the intent feature set data of the aerial target and encapsulating the domain expert knowledge and experience into labels. We improved the air target intention recognition method based on LSTM, proposed a GRU-based aerial target operational intention recognition model, and introduced a bidirectional propagation mechanism and attention mechanism to significantly improve accuracy compared to the LSTM, SAE, and DBP intention recognition models. In order to further shorten the time of air target intention recognition, we proposed the BiGRU-based air combat characteristic prediction method, and experimental results showed that it can effectively perform single-step characteristic prediction. Combining the BiGRU-Attention intention recognition module with the BiGRU characteristic prediction module, we were able to predict enemy aerial target operational intention one sampling point in advance, with 89.7% accuracy. How to more accurately distinguish confusing intentions will be our next research direction.

## Figures and Tables

**Figure 1:** Hierarchical representation and reasoning process of intention.

**Figure 2:** Schematic diagram of combat intention coding and analysis (the same color is a set of correspondences).

**Figure 3:** Relative geometric position of air combat. *H*_1_, *H*_2_ are the flight altitudes of the enemy and ours; *V*_1_, *V*_2_ are the flight speeds of the enemy and ours; D is the distance between the two parties; *ψ* is the heading angle; and *φ* is the azimuth angle.

**Figure 4:** Feature set of the tactical intention of aerial target.

**Figure 5:** Intention prediction model framework.

**Figure 6:** GRU structure.

**Figure 7:** BiGRU structure.

**Figure 8:** Attention mechanism structure.

**Figure 9:** (a) The effect of different time step on the results. (b) The effect of the number of different notes on the results.

**Figure 10:** Characteristic prediction trajectory.

**Figure 11:** Confusion matrix of intention recognition.

**Figure 12:** (a) Changes in accuracy of ablation experiment. (b) Changes in loss of ablation experiment.

**Figure 13:** (a) Changes in accuracy of four models. (b) Changes in loss of four models.

**Table 1:** Experimental results of five models.

Method	Error (10^−5^)	Prediction time (ms)
RNN	8.14	0.089
LSTM	2.75	0.133
GRU	2.46	0.110
BiLSTM	1.29	0.311
BiGRU	1.16	0.202

**Table 2:** Experimental parameters.

Parameter	Value
Loss function	Categorical_crossentropy
Optimizer	Adam
Dropout	0.5
Hidden layer	3
Hidden nodes	334, 10, 338
Batch size	100
Learning rate	0.0014
Epoch	200

**Table 3:** Comparison of model parameter settings.

Model	Number of hidden layers	Hidden notes	Learning rate	Optimizer
SAE	3	256, 128, 128	0.02	SGD
LSTM	3	256, 128, 128	0.001	Adam
DBP	4	256, 512, 512, 256	0.01	Adam

**Table 4:** Comparison of different intention recognition models.

Model	Accuracy (%)	Loss
BiLSTM-Attention	90.5	0.257
LSTM	87.6	0.346
SAE	81.3	0.473
DBP	79.3	0.492

**Table 5:** Results of ablation experiment.

Model composition structure			Accuracy (%)	Loss
Bidirectional	GRU	Attention		
√	√	√	90.5	0.257
	√	√	88.6	0.305
√	√		88.9	0.289
	√		87.4	0.337

**Table 6:** Intention prediction performance measurement.

Evaluation Index		Precision(%)				Recall (%)				F1 score			
		I	II	III	IV	I	II	III	IV	I	II	III	IV
Intent type	Surveillance	83.0	79.2	70.5	68.7	90.0	85.6	77.1	75.4	0.859	0.823	0.737	0.719
	Reconnaissance	89.9	86.8	81.0	76.3	85.3	78.8	75.4	72.4	0.876	0.826	0.781	0.743
	Feint	90.6	89.1	82.5	78.1	85.4	82.9	73.8	75.5	0.879	0.859	0.779	0.768
	Attack	82.3	79.6	71.2	70.2	90.6	89.7	81.4	73.3	0.862	0.843	0.759	0.717
	Penetration	90.3	90.0	83.4	80.8	89.9	89.6	84.9	83.1	0.901	0.897	0.841	0.819
	Retreat	97.5	98.3	93.4	95.3	94.7	93.9	91.5	91.1	0.961	0.960	0.924	0.931
	Electronic jamming	99.5	96.4	96.6	94.4	95.5	96.0	89.7	90.6	0.975	0.962	0.931	0.925

I, II, III, and IV, respectively, represent the BiGRU-Attention, LSTM, SAE, and DBP aerial target air tactical intention recognition models.

## Data Availability

The data used to support the findings of this study are available from the corresponding author upon request.
